# Radiologists versus Deep Convolutional Neural Networks: A Comparative Study for Diagnosing COVID-19

**DOI:** 10.1155/2021/5527271

**Published:** 2021-05-10

**Authors:** Abdulkader Helwan, Mohammad Khaleel Sallam Ma'aitah, Hani Hamdan, Dilber Uzun Ozsahin, Ozum Tuncyurek

**Affiliations:** ^1^Lebanese American University, School of Engineering, Department of ECE, Byblos, Lebanon; ^2^Near East University, Nicosia/TRNC, Mersin-10, 99138, Turkey; ^3^Université Paris-Saclay, CentraleSupélec, CNRS, Laboratoire des Signaux et Systèmes (L2S UMR CNRS 8506), Gif-sur-Yvette, France; ^4^University of Sharjah, College of Health Science, Medical Diagnostic Imaging Department, Sharjah, UAE; ^5^Near East University, Faculty of Medicine, Department of Radiology, Nicosia/TRNC, Mersin-10, 99138, Turkey

## Abstract

The reverse transcriptase polymerase chain reaction (RT-PCR) is still the routinely used test for the diagnosis of SARS-CoV-2 (COVID-19). However, according to several reports, RT-PCR showed a low sensitivity and multiple tests may be required to rule out false negative results. Recently, chest computed tomography (CT) has been an efficient tool to diagnose COVID-19 as it is directly affecting the lungs. In this paper, we investigate the application of pre-trained models in diagnosing patients who are positive for COVID-19 and differentiating it from normal patients, who tested negative for coronavirus. The study aims to compare the generalization capabilities of deep learning models with two thoracic radiologists in diagnosing COVID-19 chest CT images. A dataset of 3000 images was obtained from the Near East Hospital, Cyprus, and used to train and to test the three employed pre-trained models. In a test set of 250 images used to evaluate the deep neural networks and the radiologists, it was found that deep networks (ResNet-18, ResNet-50, and DenseNet-201) can outperform the radiologists in terms of higher accuracy (97.8%), sensitivity (98.1%), specificity (97.3%), precision (98.4%), and F1-score (198.25%), in classifying COVID-19 images.

## 1. Introduction

On March 1, 2020, the World Health Organization [1] declared COVID-19 as a pandemic that spread all over the world. Due to that, governments of several countries forced border restrictions and force their citizens to obey the rules of social distancing, hygiene, and wearing masks. This disease is an infection caused by a medium-sized virus characterized by its largest seen viral RNA genome [2]. Histological findings of COVID-19 are characterized by an acute and organizing diffuse alveolar damage [3].

As for now, COVID-19 is still a global crisis, it has killed at least 715 thousand people worldwide at the time of writing this paper in the first week of August 2020, and it caused the death of more than 2.82 million people at the time of the last pre-publication reading of this paper on April 3, 2021.

Despite the discovery of effective vaccines for COVID-19 [4], it remains important to diagnose this disease accurately. The diagnosis tool that has been employed since the breakthrough of COVID-19 has mainly been the real-time reverse transcriptase polymerase chain reaction (RT-PCR). RT-PCR or PCR for short is used to detect the nucleic acid of the virus in the upper and lower respiratory specimens [5]. Such diagnosis tool, however, was seen to be insufficient for this highly contagious and rapidly spreading disease, as it showed a sensitivity ranging between 37% and 71% according to some early reports [6–8].

Chest computer tomography (CT) and X-rays started to be investigated as additional tools for diagnosing COVID-19 due to their observed effects on the lungs in a significant number of individuals. In March 2020, datasets consisting of chest CT and X-ray images of healthy as well as COVID-19-infected individuals started to be uploaded to many data repositories such as GitHub and Kaggle. Since then, researchers started to investigate the efficiency of deep learning in classifying COVID-19 and Non-COVID-19 chest CT and X-ray images. Afterwards, many related studies were proposed such as differentiating COVID-19 from other viral pneumonias [9], and comparison of COVID-19 chest CT diagnosis sensitivity with RT-PCR [10].

In this study, our aim is slightly different, as it is not to compare between automated COVID-19 diagnosis methods, but rather it is to compare the performance, in terms of COVID-19 diagnosis, of humans (Radiologists) to the performance of machines deploying automated deep learning-based methods. We aim to investigate the generalization capabilities of both radiologists and deep learning networks in diagnosing COVID-19 and differentiating it from other chest diseases. Hence, we tested both radiologists and deep learning methods using a test set of 250 images of COVID-19 and Non-COVID-19 cases to compare their generalization power in diagnosing COVID-19. The results show that the radiologists failed to compete with deep learning networks in which networks achieved higher accuracy, sensitivity, specificity, precision, and F1-score than those achieved by the radiologists when tested on a small test set of images. This outperformance is discussed throughout the paper and explained in the Results and Discussion section. The paper is organized as follows: Section 1 is an introduction of the paper.  Section 2 is a review of some papers discussing deep learning versus humans' performance comparison.  Section 3 discusses the dataset, networks used, and selection of radiologists for this paper.  Section 4 shows the transfer learning and evaluation metrics used in evaluating the deep learning networks.  Section 5 is about the results of training and testing deep learning networks and radiologists. Finally, Section 6 is a conclusion of the whole work.

## 2. Related Works

Due to the success and rapid deployment of deep learning methods and architectures, humans are keen to compare the performance of deep learning-based systems to their own. Human versus machine comparison studies in medicine are several. However, for COVID-19 as a case study, such studies are very limited as COVID-19 is a recent disease. In this section, we review some studies that compare the medical experts and deep learning's diagnosis capabilities in general medicine.

### 2.1. Medical Experts versus Deep Neural Networks (DNNs) in Medicine

In 2017, a group of researchers proposed a deep network for the classification of skin cancer [11]. The authors used an end-to-end convolutional neural network (CNN) that was trained using image pixels and labels as inputs and outputs, respectively. In their study, the performance of the trained CNN was tested against 21 board-certified dermatologists and it was found that the CNN can perform on par with all certified experts. This demonstrated that a neural network is capable of classifying skin cancer with a good human level of competence.

Moreover, a systematic review and meta-analysis was proposed by a group of authors in order to study the performance of health-care professionals versus deep learning methods in detecting different diseases [12]. This study scrolls over 31587 articles that compare the performance of medical professionals versus deep learning performance in specific medical classification tasks. Only the well-reported studies that discuss the accuracy, sensitivity, specificity, and other DNN's evaluation metrics were selected to be part of this study, as claimed by the authors. Experimentally, it was found that the performance of deep learning models is equivalent to that of the health-care professionals in most of the studies of medical classification tasks. Moreover, another major finding of this related work is that the studies, which validated or tested the deep learning models on the same samples or images that were used to assess the performance of the health-care professionals, were very few. In contrast, in our study, we tend to test the radiologists and CNNs using the same chest CT images to ensure a fair comparison.

### 2.2. Human versus DNN in Medicine: COVID-19 as a Case Study

To our knowledge, there is only one recent published research by Mei et al. (2020) about the comparison of the radiologists versus deep learning performance for chest CT COVID-19 and other clinical attributes such as symptoms, history, and laboratory testing [13]. The work of Mei et al. [13] is an integration of the chest CT and the afore-mentioned attributes for the rapid diagnosis of COVID-19. Three different neural network models were used, consisting of a CNN, MLP (multilayer perceptron), and a joint model which is described by the authors as a combination of a CNN and a MLP joined together to diagnose COVID-19 using medical imaging (CT) and clinical attributes. The performance of the trained models is compared to the performance of a senior thoracic radiologist and a thoracic radiology fellow. It was found that, for new and unseen images, the joint model gained more powerful generalizing capability than that achieved by the radiologists, in terms of area under curve (AUC). As a result, despite the limitations of this study discussed in Section 5, it yet demonstrates a good capability of deep learning in outperforming the medical experts in diagnosing chest CT COVID-19.

In our work, we aim to employ state-of-the-art deep neural networks in medical applications for the purpose of classifying chest CT images into COVID-19, Non-COVID-19, and tumor. Additionally, we aim to compare the performance of the considered deep neural networks to the performance of junior and senior radiologists in terms of their capabilities of diagnosing the same test images, and to derive some findings.

## 3. Materials and Methods

Chest CT image datasets, state-of-the-art deep neural networks, and medical experts, were all the requirements for this study. In this section, the constructed and employed dataset is described, in addition to the deep convolutional neural networks that were employed in this work to perform the COVID-19 diagnosis task. Moreover, the radiologist's experimental procedure of receiving and diagnosing the chest CTs is also explained.

### 3.1. Dataset

In this study, after securing the ethics committee's approval (2020/85-1187), a dataset was constructed consisting of 3000 chest CT images. The chest CT images were collected from the PACS system of the Department of Radiology associated with the Near East University Hospital [14].

The dataset includes images of two different classes: COVID-19 (positive) and Non-COVID-19 (negative). Note that the COVID-19 class means that a patient is positive for the Coronavirus no matter what other chest diseases are found. Non-COVID-19 indicates that a patient is negative for the Corona disease; however, this does not necessarily mean that the CT is normal, as it may have other bacterial or other types of viral pneumonias. The patients who underwent thorax CT between January 2020 and March 2020 were evaluated retrospectively. The CT images of the patients were obtained using a Siemens Somatom Definition Flash (Erlangen, Germany) machine. FOV: 380 mm, Slice thickness: 1 mm, mAs: 70, and kV: 120, were used with the thorax CT protocol.

The data collected is comprised of 1500 COVID-19 and 1500 Non-COVID-19 images.  Table 1 shows how the data is split into training, validation, and testing.  Figure 1 shows a sample of COVID-19 and Non-COVID-19 images from the dataset.

Note that we used a small validation set as we are applying transfer learning; hence, few hyperparameters need to be fine-tuned. Moreover, test set was also small for some reasons explained in the Discussion section.

### 3.2. Deep Neural Networks

Deep convolutional neural networks invaded the image classification world due to their very high accuracies in classifying natural images, when trained on huge amounts of images found in big benchmark datasets such as ImageNet [15]. Hence, researchers started to use such pre-trained deep neural networks for different classification purposes such as medical image classification [16]. The most efficient technique to retrain a deep network, that is already trained using ImageNet, is transfer learning. This technique allows the network to be trained to perform a new classification task that is different than its primary classification one by fine-tuning some of the deep neural networks' parameters and freezing others [17].

Recently, researchers started to apply transfer learning to different pre-trained models in order to perform a new classification task such as the task of COVID-19 detection or diagnosis. In this context, several deep neural networks were employed for different classification paradigms. Some studies aimed to classify COVID-19 (positive or negative) [18–21] while others attempted to distinguish the COVID-19 infection from other bacterial and viral infection [22]. In most of these prior studies, the datasets that were used to train and test the employed deep neural networks are either chest X-ray or chest CT images. However, in our study, we focus on chest CT images; therefore, we will only discuss the studies that use chest CT images to train their models.  Table 2 shows some studies that employed deep convolutional neural networks to classify or detect COVID-19 using chest CT images. We selected state-of-the-art CNNs that scored the highest accuracies in correctly classifying COVID-19.

As it can be seen from Table 2, ResNet-18, ResNet-50, and DenseNet-201, achieved the highest accuracies in detecting COVID-19; thus, in our study, we used the same three networks' structures and we applied transfer learning to retrain these models using our dataset. The deep neural networks are then tested using a set of images (testing image set), that are not part of the training image set nor part of the validation image set. Furthermore, in order to compare the deep neural networks' performance to the human performance, this same testing image set is used by the radiologists for diagnosis.

### 3.3. Medical Experts Selection

Neural networks were developed as an attempt to mimic the human brain functionality. They both have interconnected neurons that transmit information to correlate input and output messages or signals [23]. For humans, learning is acquired from experience which is the knowledge acquired during the time spent on learning and performing a certain task. For a neural network, experience is the number of examples used for training and fine-tuning. Hence, the analogy of neural network to human experience is that several years of experience for humans (seniors) are considered as training the network on huge amounts of images. On the other hand, training a neural network using a relatively small number of images can be seen to be analogous to only few years of experience for humans (juniors), in case of human to machine comparison.

In our case, the used dataset is relatively small as compared to ImageNet. However, it is of average size when compared to datasets for fine-tuning pre-trained models. Hence, we selected two types of medical experts: one is a thoracic radiologist with 10 years of experience in thoracic imaging (Rad 1) and the other is a junior radiologist with 2 years of experience in the same field (Rad 2). It is also important to mention that these radiologists' main experience has been in chest X-ray diseases diagnosis such as pneumonia, effusion, mass, etc. As for COVID-19, most radiologists have no more than one-year experience in COVID-19 diagnosis (since the onset of the COVID-19 pandemic), except that some radiologists may have encountered more Coronavirus infected cases than others.

Images were selected randomly from the dataset to form the testing set to be sent to the radiologists for diagnosis, with 100 and 150 images randomly selected from the COVID-19 and Non-COVID-19 classes, respectively. A deadline of 14 hours was set as the time required to finish diagnosing all images. It should be noted that this time period was selected by a senior radiologist as an adequate time period for such number of images to be diagnosed by radiologists. Both radiologists respected the set time and submitted their diagnosis results within the requested time period.

## 4. Transfer Learning

### 4.1. Transfer Learning

We adopted three different pre-trained deep neural networks named as: ResNet-18 [24], ResNet-50 [24], and DenseNet-201 [25]. These models are called pre-trained models as they were initially trained on large benchmarks to solve some image classification tasks. In order to use these models for our new task (COVID-19 diagnosis from chest CT images), we use the transfer learning approach. This approach is popular in deep learning as it enables the model to be trained faster by starting with initial patterns and parameters that were learned in a different classification task. To start the training process using transfer learning, we used the predefined and pre-trained weights and filters for every employed CNN, which were slightly updated during the learning process for the classification of COVID-19 and Non-COVID-19. More details about the learning process are provided in Section 5.1.

For our collected data acquired, the images were first converted from the Digital Imaging and Communications in Medicine (DICOM) format to the three-channel PNG format. As for preprocessing, images were only normalized to scale their pixel values to the range of 0 to 1 and resized to 224 × 224 pixels to fit the employed models' inputs.

Figure 2 illustrates the adopted transfer learning-based scheme to classify COVID-19 and Non-COVID-19. As it can be seen from Figure 2, we removed the classification part (i.e., part consisting of the fully connected layers) of the pre-trained models and replaced it with a new classifier that consists of two output classes: COVID-19 and Non-COVID-19. The role of this classifier is to classify images based on the activations it receives from the feature extraction part of every CNN. The activations are first flattened, and then, two fully connected (FC) layers are added. The first FC layer consists of 32 nodes while the second one consists of 2 nodes, representing the two different classes. Finally, the two different activations of the second FC layer are fed into a Softmax layer that produces the probability of each class (COVID-19 and Non-COVID-19). The class with the highest probability is chosen to be the final predicted class.

### 4.2. Evaluation Metrics

The fine-tuned deep neural networks are evaluated by calculating their testing accuracies as given below:

(1) $$\begin{array}{c} \text{Accuracy}=\frac{N}{T}, \end{array}$$

where *N* is the number of correctly classified images, while *T* represents the total number of images.

In addition to the accuracy metric, more evaluation metrics, such as sensitivity, specificity, precision, and F1-score, are also used to evaluate the fine-tuned models as well as the radiologists:

(2) $$\begin{array}{c} \begin{array}{c} \text{Sensitivity}=\frac{\text{TP}}{\text{TP}+\text{FN}}, \end{array}\\ \begin{array}{c} \text{Specificity}=\frac{\text{TN}}{\text{TN}+\text{FP}}, \end{array}\\ \begin{array}{c} \text{Precision}=\frac{\text{TP}}{\text{TP}+\text{FP}}, \end{array}\\ \text{F}1\text{‐score}=2*\frac{\text{precision}*\text{sensitivity}}{\text{precision}+\text{sensitivity}}, \end{array}$$

where TP stands for true positive, and it indicates the number of correctly predicted positive classes (i.e. COVID-19); TN stands for true negative, and it indicates the number of correctly predicted negative classes (i.e. Non-COVID-19); FP refers to false positive, and it indicates the number of incorrectly predicted positive data samples, while FN is the false negative, and it indicates the number of incorrectly predicted negative data samples.

## 5. Results and Discussion

### 5.1. Network Fine-Tuning

The networks were all implemented using the Keras library, the official front end of TensorFlow. As stated previously, the networks were trained to perform the COVID-19/Non-COVID-19 classification task via transfer learning, wherein the training set of our dataset (see Table 1) was used to fine-tune pre-trained network models. The pre-trained networks were fine-tuned using a categorical cross-entropy cost function and stochastic gradient descent (SGD) with a small learning rate of 0.0001 and a batch size of 64 on a GeForce GTX 1640Ti graphical processing unit (GPU). A small validation set of 133 images (see Table 1) was used to validate the networks and to further fine-tune their parameters. The training and validation image sets were randomly shuffled in order to have shuffled batches to avoid images correlation.

The number of training epochs is selected based on the variations of the accuracy and validation error [26, 27]. This is achieved by monitoring the validation error of each of the considered networks as it can be associated with optimization problems, i.e., if it is high, overfitting may occur. In our implementation, a maximum number of 10 epochs was selected, and the deep neural networks were allowed to stop learning once the validation error started to increase, and/or the accuracy started to saturate.

Figure 3 shows the learning curve and loss of deep convolutional neural networks. It is seen that all models achieved significant accuracies during training. However, ResNet-50 required a greater number of epochs than the other networks in order to reach its highest training accuracy. This may be because of its depth and most importantly its huge number of learnable parameters.

### 5.2. Testing and Comparison

The resulting fine-tuned deep neural networks (DNNs) were tested on the dataset's testing image set consisting of 250 images: 100 images from the COVID-19 class and 150 from the Non-COVID-19 class (see Table 1). Moreover, these same images were used to test the radiologists' capabilities to diagnose images as COVID-19 or Non-COVID-19. The performance of the deep neural network models and the radiologists in relation to diagnosing COVID-19 is summarized in Table 3.

From Table 3, it can be seen that the fine-tuned deep neural network models show good generalization capabilities in the sense that these models reached relatively high accuracies when tested on new and different COVID-19 and Non-COVID-19 images, instead of those used in training and validation. More specifically, DenseNet-201 achieved the highest accuracy (97.8%) among all the employed deep neural networks. This may be due to its depth as it is deeper than all other employed deep neural networks. The larger depth allows DenseNet-201 to extract more abstract and distinguishable features, which helps in more accurate diagnosis. DenseNet-201 consists of more layers as compared to ResNet-18 and ResNet-50. Hence, the DenseNet-201 network has the capacity of learning a larger number of parameters as compared to ResNet-18 and ResNet-50 due to its larger depth. This allows it to extract latent space features that help in classifying COVID-19 from Non-COVID-19 more accurately. DenseNet-201 contains more than 18 million learnable parameters, which allows it to create an abstract representation of input images to reach a very high classification rate. On the other hand, it is seen that ResNet-50, which has a larger number of learnable parameters as compared to DenseNet-201, still could not beat the DenseNet-201 in terms of accuracy. This, however, makes the ResNet-50 train slower with more computation cost, as compared to ResNet-18 and DenseNet-201 (see Figure 3). Table 3 shows also that ResNet-18 achieved the lowest generalization capability as compared to the other employed deep neural network models. This is expected because of its depth, as it contains only 18 layers which make its training faster than that of ResNet-50, whereas its performance is poorer.

Moreover, Table 3 shows the performance of the two radiologists in classifying COVID-19 and Non-COVID-19 images. The first radiologist (Rad 1) achieved a higher accuracy (76.4%) than the second one (Rad 2) who reached an accuracy of 75.9%. It is also seen that the other metrics (sensitivity, specificity, precision, and F1-score) are also higher for Rad 1 as compared to Rad 2. This outperformance by Rad 1 over Rad 2 is possibly because of the experience that Rad 1 has over Rad 2, as he/she is a senior radiologist with 10 years of experience in thoracic imaging and exploring different chest diseases.

It is also noticeable, in Figure 4, that all employed deep neural network models outperformed the medical experts' diagnosis (Rad 1 and Rad 2) in terms of accuracy as well as the other performance metrics (see Table 3). This outperformance of deep learning over human experts can be due to several reasons. The most common one is that COVID-19 is a recent disease, and radiologists may have not seen many related chest CTscans; hence, they still have not gained sufficient experience in diagnosing COVID-19 accurately, and differentiating it from other classes and conditions, in particular, pneumonia. One more reason may be the lack of enough knowledge about the Coronavirus and how it manifests itself on a chest CT.  Figure 5 shows the receiver operating characteristic (ROC) curve of the DenseNet-201.

For a better interpretability of the employed model that achieved the highest accuracy on the testing data (DenseNet-201), we visualize the gradient weight class activation mapping (Grad-Cam) of some correctly classified testing images. This method enables one to visualize the activations in the areas that the deep neural network focused on to classify a certain image. The suspected regions associated with a predicted class are highlighted using heatmaps, in which a jet colormap shows the highest activation regions as deep red, and the lowest activation regions as deep blue.  Figure 6 shows the Grad-Cam of some testing images that were correctly classified by DenseNet-201.  Figure 6(a) shows the COVID-19 examples, while Figure 6(b) shows the Non-COVID-19 images. The deep red in Figure 6 shows the regions that have the highest activations which the model relies on to classify an image. It is noted that for the COVID-19 examples, the heatmap indicated large intensities over several regions in both images.

### 5.3. Discussion

In this study, we showed that a deep artificial neural network can outperform a radiologist in diagnosing COVID-19 and in distinguishing COVID-19 from other Non-COVID-19 cases. The basic idea is that our transfer learning based deep neural network (DenseNet-201) was trained on 2617 images (see Table 1). However, we are not sure about the number of COVID-19 images that the radiologists have seen, as COVID-19 is a recent disease and the radiologists have not yet seen all its aspects. On the other hand, we believe that our selected radiologists already have significant experience with various chest diseases which can help them in differentiating these from the COVID-19 virus disease.

One can also attempt to train the radiologists on the same images that were used for training the networks by displaying them correspondingly with their true labels, for a short period of time. However, such training would be very time consuming for the radiologists and therefore would not be feasible. Thus, there was a need to reduce the number of images selected for testing the radiologists as much as possible. Consequently, the number of images used for testing the deep neural network models was also small, as the same images were used for testing the performance of both the radiologists and the deep neural network models. Testing the deep neural network on a larger number of images (e.g. 50% of the whole data) may change the results. Therefore, we tested our trained DenseNet-201 on another dataset of chest CT COVID-19 and Non-COVID-19 [28]. This dataset was evaluated and confirmed by a senior radiologist from Tongji Hospital, Wuhan, China. The dataset contains 300 images of COVID-19 and 300 images of Non-COVID-19, and they were all used to test the DenseNet-201; the result is shown in Table 4.

As it can be seen from Table 4, the deep neural network's performance decreased when tested on another dataset, which contains more testing images and different characteristics than ours such as quality of images. The aim of testing the network on another dataset that was not seen before, and that contains many testing images, is to show that the DenseNet-201's performance may decrease when testing ratio increases and to make a fair comparison with radiologists.

## 6. Conclusion

In this study, ResNet-18, ResNet-50, and DenseNet-201, were investigated for the diagnosis of COVID-19. Transfer learning approach was applied on these three pre-trained deep neural network models to perform one more additional classification task. Moreover, this work aims to compare the medical radiologists COVID-19 diagnosis skills with that of the pre-trained deep neural networks that are fine-tuned on 2617 chest CT images of COVID-19 and Non-COVID-19. A test set of 250 images was diagnosed by the deep neural network models and the radiologists, and as a result, it was observed that DenseNet-201 outperformed all the other investigated deep neural networks in terms of overall accuracy. Furthermore, it was also observed that all the investigated deep neural network models have outperformed the two radiologists in correctly diagnosing the COVID-19 chest CT images. This outperformance of deep learning over medical experts does have some limitations discussed in the Discussion section. Nevertheless, for a better conclusion, a larger amount of data can be used to train and, most importantly, to test the deep neural networks and the radiologists, and to derive more abstract findings.

## Figures and Tables

**Figure 1:** Samples of the chest CT image dataset.

**Figure 2:** Scheme of transfer learning-based networks for the classification of COVID-19 and non-COVID-19.

**Figure 3:** Accuracies and losses reached by every model during training.

**Figure 4:** Comparison of deep neural network models and radiologists in terms of COVID-19 diagnostic accuracy.

**Figure 5:** ROC curve of the DenseNet-201.

**Figure 6:** Activation maps (Grad-Cam) of the predicted classes of the DenseNet-201.

**Table 1:** Chest CT image dataset description.

	Total number of images	Training	Validation	Testing
COVID-19	1500	1317	83	100
Non-COVID-19	1500	1300	50	150

**Table 2:** State-of-the-art deep neural networks for diagnosing COVID-19 from chest CT images.

Authors and year	Deep network	Classes	Performance metrics (overall accuracies)
Wang et al., (2020) [18]	DeCovNet	COVID-19 and non-COVID-19	90.1%
Singh et al., (2020) [19]	ResNet-18	COVID-19 and non-COVID-19	99.4%
Ahuja et al., (2020) [20]	MODE-based CNN	COVID-19 and non-COVID-19	93.3%
Jaiswal et al., (2020) [21]	DenseNet-201	COVID-19 and non-COVID-19	97%
Ko et al., (2020) [22]	ResNet-50	COVID-19, pneumonia, nonpneumonia	96.97%

**Table 3:** Performance metrics of the employed deep neural network models and the radiologists on the testing images.

	Accuracy	Sensitivity	Specificity	Precision	F1-score
Rad 1	76.4%	79.1%	80.3%	80.4%	79.74%
Rad 2	75.9%	74.1%	78.7%	79.2%	76.56%
ResNet-18	91.3%	90.1%	94.3%	91.4%	90.74%
ResNet-50	97.2%	93.1%	94.3%	96.1%	94.58%
DenseNet-201	97.8%	98.1%	97.3%	98.4%	98.25%

**Table 4:** Testing DenseNet-201 on a new dataset.

	Number of testing images	Accuracy
Dataset 1 (ours)	250	97.8%
Dataset 2	600	65.3%

## Data Availability

Correspondence and requests for materials and data should be addressed to Helwan, A.
